# Grass-Shaped Zinc Oxide Nanoparticles Synthesized by the Sol-Gel Process and Their Antagonistic Properties towards the Biotrophic Parasite, *Meloidogyne incognita*

**DOI:** 10.1155/2023/6834710

**Published:** 2023-03-24

**Authors:** Amir Khan, Azmat Ali Khan, Mohd Jameel, Mohd Farhan Khan, Masudulla Khan, Arshad Khan, Faheem Ahmad, Mahboob Alam

**Affiliations:** ^1^Department of Botany, Aligarh Muslim University, Aligarh 202002, India; ^2^Pharmaceutical Biotechnology Laboratory, Department of Pharmaceutical Chemistry, College of Pharmacy, King Saud University, Riyadh 11451, Saudi Arabia; ^3^Department of Zoology, Aligarh Muslim University, Aligarh 202002, India; ^4^Department of Science, Gagan College of Management and Technology, Aligarh 202001, India; ^5^Botany Section, Women's College, Aligarh Muslim University, Aligarh 202002, Uttar Pradesh, India; ^6^Department of Safety Engineering, Dongguk University, 123 Dongdae-ro, Gyeongju-si, Gyeongbuk 780714, Republic of Korea

## Abstract

The presence of *Meloidogyne* spp., also known as root-knot nematodes, presents a significant danger to global agricultural progress. Since chemical nematicides have high levels of toxicity, it is imperative to develop environmentally friendly methods to manage root-knot nematodes. Nanotechnology is now the most progressive way to attract researchers due to its innovative quality in combating plant diseases. Our study focused on the sol-gel process to synthesize grass-shaped zinc oxide nanoparticles (G-ZnO NPs) and assess its nematicidal behavior against *Meloidogyne incognita*. Various concentrations (250, 500, 750, and 1000 ppm) of G-ZnO NPs were utilized to expose both the infectious stage (J2s) and egg masses of *M. incognita*. Laboratory results revealed that G-ZnO NPs showed toxicity to J2s with LC50 values of 1352.96, 969.64, and 621.53 ppm at 12, 24, and 36 hours, respectively, and the result was the inhibition of egg hatching in *M. incognita*. All three exposure periods were reported linked with the concentration strength of G-ZnO NPs. The pot experiment results exhibited that G-ZnO NPs significantly reduced the root-gall infection of chickpea plants under *M. incognita* attack. Compared with the untreated control, there was a significant improvement in plant growth attributes and physiological parameters as well, when distinct G-ZnO NP doses (250, 500, 750, and 1000 ppm) were applied. In the pot study, we noticed a reduction in the root-gall index with an increase in the concentration of G-ZnO NPs. The results confirmed that G-ZnO NPs have enormous potential in sustainable agriculture for controlling the root-knot nematode, *M. incognita*, in chickpea production.

## 1. Introduction

Pulses are the richest source of protein and play an important role in vegetarian diets. India is a major pulse-growing country globally, accounting for 35–36% of the area and 27–28% of the production [1]. Chickpea (*Cicer arietinum* L.) is the second most grown pulse crop across the globe, occupying 14.6 million acres [2]. However, chickpea production is remarkably affected due to pests and diseases [3]. According to Bhatti [4–6], plant-parasitic nematodes (PPNs), including RKNs, parasitize chickpea plants and constrain the yield. The RKN, *M. incognita*, is the most widely distributed species responsible for most crop losses, including chickpeas [7, 8]. Farmers and agriculturists have long used chemical pesticides to manage the RKN population below a threshold successfully. The reason behind choosing it is because of its immediate effects on RKNs. However, these chemicals are prohibited and not recommended in most countries because of their adverse impacts on the environment and human and animal health [9]. Keeping the harmful effects of chemical pesticides in mind, researchers focusing on alternative cost-effective, environmentally friendly, and safe options for controlling pests and diseases, including nematodes disease, have become a concern. Sustainable options, such as beneficial microorganisms, biopesticides, natural plant products, and biocompatible nanopesticides were used to combat pests and diseases, such as root-knot nematodes [10–15]. Nanotechnology is a multidisciplinary field of study that has the potential to transform the agricultural landscape in terms of plant disease control, pathogen recognition, and pesticide degradation [6, 16]. Due to low environmental impacts, the utilization of NPs in agriculture has grown in prominence over the last few decades [17]. In the scientific literature, several preparation methods, such as the sol-gel approach, solution-precipitation approach, spray-pyrolysis, hydrothermal approach, microwave-assisted technique, and water-assisted synthesis, have been explored. These methods have produced ZnO NPs in a variety of shapes and sizes, including nanothorns, nanorods, nanoflowers, nanopillars, nanograss, microspheres, and nanoprisms [18]. Once applied to soil, the particles slowly release the compound where necessary and limit uncontrolled spreading into subsoil with rain and irrigation. Moreover, using biodegradable nanoparticles avoids any potential risk associated with residual, synthetic nanomaterials in the subsoil, which is typical of other nanopesticides based on nonbiodegradable carriers. Compared with nanoparticle-assisted fabrications of nanostructures, nanograss has a better size uniformity. Abdellatif et al. [19] investigated the effect of silver nanoparticles (AgNPs) on the reproduction and development of *M. javanica* and showed that AgNP application was uniformly efficient as chemical behavior in lowering egg masses per root system. In their study, Khan et al. [6, 20] found that treatment with CuO nanoparticles enhanced growth and physiological attributes of cowpea and chickpea and decreased galls, egg masses, and the J2s population of *M. incognita*. The potential of green-produced ZnO NPs as a nano-based agricultural fertilizer foundation has been explored [21]. Thus, our study focused on a cost-effective and straightforward sol-gel technique to produce the G-ZnO NPs for the antagonistic activity. So, it would be utilized as a nano-based fertilizer source in agriculture. In the current study, using the sol-gel technique, zinc acetate dihydrate and sodium hydroxide were combined in presence of a cationic surfactant, palmityl trimethyl ammonium bromide, to produce G-ZnO NPs. Furthermore, antagonistic efficiency was tested against RKN, *Meloidogyne incognita*.

## 2. Materials and Methods

### 2.1. Materials

The chemicals, including the ion-carrier sodium hydroxide, zinc acetate dihydrate, and the capping agent, palmityl trimethyl ammonium bromide, were of analytical quality and obtained without additional purification from E. Merck Limited (Mumbai, India) and Loba (Mumbai, India). The glassware was purchased from Borosil in India. Throughout the experiments, double-distilled water (DDW) was utilized. In this study, chickpea and RKN, *M. incognita*, were used as test plants and pathogens, respectively. Infected brinjal roots were used to harvest egg masses of *M. incognita* in order to produce second-stage juveniles (J2s) for hatching.

### 2.2. Synthesis of G-ZnO NPs

The sol-gel process was utilized to synthesize the G-ZnO NPs. A total of 0.135 gm of zinc acetate dihydrate, 1.767 gm of palmityl trimethyl ammonium bromide, and 0.219 gm of sodium hydroxide were taken and gradually dissolved in 100 mL DDW separately. Henceforth, the mixed solution of palmityl trimethyl ammonium bromide and zinc acetate dihydrate taken in a flat-bottomed flask is vigorously agitated during the experiment. In continuation, the sodium hydroxide solution is dispensed into the flask drop by drop, eventually leading to completion. After a few minutes, the ambiguous droplets with a thick frothy layer on top of the colloidal suspension could be seen in the flask, which is maintained at a constant temperature, namely, ambient. The resulting dispersion liquid is cooled for some time before being centrifuged, cleansed, and stored for further characterization after adequate drying.

Previously, our team produced flower-shaped ZnO NPs at varying temperatures utilizing a simple sol-gel synthesis method without the need for complex equipment [22]. In addition, we looked at how mechanical stirring affected the formation of thorn-shaped ZnO NPs during their synthesis [23]. Under this work, the diverse growths of long grass-likeone-dimensionalG-ZnO NPs crystals were achieved with the help of the sol-gel method on extending the incubation duration after synthesis while maintaining a constant temperature. We developed G-ZnO NPs crystals and discovered that they improved chickpea growth and production while also reducing *M. incognita* infection. In combination with all, the study showed that in vitro J2s hatching of *M. incognita* was inhibited by NPs, which also caused J2s mortality, suggesting their utility in the biological management of *M. incognita*. Moreover, a study demonstrated the usefulness of G-ZnO NPs on various plant development metrics grown in nematode-infected soil.

### 2.3. Collection and Growth of *M. incognita* Inoculum (J2s)

The pure population of *M. incognita* was maintained in the glasshouse of the Department of Botany at Aligarh Muslim University (India) using infected brinjal roots. The perineal pattern was used to determine whether *M. incognita* was present [24]. Bogner's approach was used to extract the nematode eggs [25]. Fresh roots were washed and cut into 1 cm pieces before being immersed for 5 minutes in a 0.6% (w/v) sodium hypochlorite solution and sonicated. After being washed 3 times with DDW, the pieces were sieved using 200 mesh and 500 mesh screens. The eggs were collected at the sieve's bottom with a mesh size of 500. The eggs were collected and kept in the BOD incubator at 27°C ± 2 on Petri dishes with DW. On a daily basis, the suspension consisting of hatched J2s was gathered, and additional DDW was introduced. The concentration of newly hatched J2s was determined and utilized for subsequent investigations.

## 3. *In Vitro* Analysis

### 3.1. Mortality Test

The nematicidal activity against J2s was tested using different concentrations (250, 500, 750, and 1000 ppm) of G-ZnO NPs, and for each treatment, the LC_50_ value was calculated. 1.5 ml of DW containing 110 newly hatched J2s was put into Petri plates with 8.5 ml of a concentration of 250, 500, 750, and 1000 ppm to examine the effect of G-ZnO NPs on J2s mortality. Petri dishes only containing DDW were employed as a control. To prevent evaporation and J2 mortality, the Petri plates were covered with Parafilm and the J2s were examined for mortality at 12, 24, and 36 hours using a dissecting microscope. Each treatment was replicated five times. If nematodes moved or twisted, they were considered living [26]. If they did not start moving again after being put in tap water and punched with a needle, they were considered dead [27]. Probit analysis was used to obtain the LC_50_ value of every treatment based on concentrations and percent mortality data [28, 29]. The percentage mortality was found employing the rule given below.

(1) $$\begin{array}{c} Percent\;mortality=\frac{C0-T\alpha }{C0}X100\text{,} \end{array}$$

where C0 = count of active J2s in the control; T*α* = number of active J2s after 12 hours, 24 hours, and 36 hours of exposure to various concentrations of G-ZnO NPs.

### 3.2. Hatching Bioassay

Inhibitory effects of G-ZnO NPs on J2s hatching at various concentrations (250, 500, 750, and 1000 ppm) were examined using the dipping technique. Five egg masses of *M. incognita* have been handpicked with forceps, from roots of infected brinjal, and 10 ml of G-ZnO NPs at the abovementioned concentrations were placed in Petri plates. To prevent evaporation, wrapped in parafilm, Petri dishes were incubated at 28°C. As a control, egg masses were immersed in DDW. Each treatment, except for the control, was done five times. After three days, the number of hatched J2s in each replicate is counted using a binocular microscope to determine the hatching values for each replicate. Then, the following formula is used to figure out the percent inhibition of egg hatching in each replicate [30].

(2) $$\begin{array}{c} Percent\;inhibition\;in\;J2s\;hatching=\frac{Number\;of\;J2s\;hatched\;in\;control-Number\;of\;J2s\;hatched\;in\;each\;concentration}{Number\;of\;J2s\;hatched\;in\;control}\times 100\text{.} \end{array}$$

### 3.3. Infectivity Bioassay (Pot Study)

In this experiment, the pathogenicity rate was measured using a pot study in a glasshouse. Susceptible chickpea cv. Avrodhi was used to evaluate the nematotoxic potential of G-ZnO NPs against *M. incognita* at various concentrations (250, 500, 750, and 1000 ppm). The clay pots with a diameter of 15 centimeters were each filled with 1 kg of autoclaved soil at a proportion of 3 : 1 (sandy loam: farmyard manure). Chickpea seeds were sterilized and sowed in each pot after being exposed to 1.0% sodium hypochlorite (NaOCl) for 15 minutes. After two weeks, one normal and vigorous seedling was kept in every treated pot, while the remaining were removed from the ground level.

### 3.4. Experimental Design

This research was carried out in a completely randomized block, with 5 replicates for each treatment, including control. Treatments include the following: (a) healthy control (without J2s and G-ZnO NPs), (b) nematode inoculated control (J2s only), (c) pot treated with 10 ml of 250 ppm of G-ZnO NPs, (d) pot treated with 10 ml of 500 ppm of G-ZnO NPs, (e) pot treated with 10 ml of 750 ppm of G-ZnO NPs, and (f) pot treated with 10 ml of 1000 ppm of G-ZnO NPs. Approximately 2,500 J2s were inoculated close to the root zone by creating 10 mm holes and then holes filled with sterilized soil. Plants were irrigated respectably during the experiment and with care to avoid examination errors. After 60 days, plants were taken out and rinsed with running tap water to take away adhering soil particles. Several growths, physiological, and pathological parameters are also taken into consideration.

### 3.5. Determination of Growth, Yield, and Physiological Parameters

In consideration of growth measurements, photosynthetic pigments (chlorophyll and carotenoid content (mg/g)) were measured by Mackinney [31] and MacLachlan and Zalik [32], respectively.

### 3.6. Determination of Pathological Parameter (J2s Population)

Cobb's sieving and decanting method [33] has been utilized to calculate the final J2s population of *M. incognita* in the soil at the time of harvesting, followed by a modified Baermann's funnel technique [34].

### 3.7. Characterization of G-ZnO NPs

#### 3.7.1. X-Ray Diffraction (XRD) of G-ZnO NPs

The X-ray diffraction of synthesized G-ZnO NPs was performed using an AXD D8 ADVANCE BRUKER (Germany) X-ray diffractometer with a nickel filtered copper K*α* radiations with wavelength 1.54 Å including scale dimensions of 0.01° with scanning speed of 0.02 scales per second. The power production is set at 40 kV and 40 mA. The Debye–Scherer formula [35, 36] is used to compute the nano-particulate sizes using spectral peaks:

(3) $$\begin{array}{c} D=\frac{k\lambda }{\beta \;\cos\;\theta }\text{,} \end{array}$$

where *D* = Size of crystallite. *k* = 0.9 (Proportionality constant). *λ* = 1.54178 Å (applied X-ray wavelength). *β* = FWHM of XRD peaks. *θ* = Braggs' angle.

The embedded application, the Diffrac plus, makes the computation easier.

The dimension of G-ZnO nanoparticles was determined using a transmission electron microscope (TEM) with rapid collecting data and ultrahigh resolution. G-ZnO NPs have been lyophilized and suspended in 20 mM phosphate-buffered saline (PBS, pH 7.4). A drop of NPs was deposited on a transparent glass shaft, let air dry in the air, and then coated using a sputter coater with a gold-palladium composite material. For imaging purposes, a 200 kV accelerating voltage was used [37]. The surface characterization of G-ZnO NPs was analyzed using SEM with JEOL JSM-6510 LV (Japan) by measuring the proportion of the morphological aspect (shape and d/l values). This study was coordinated by Oxford's EDS and SEM. The samples were examined through an accelerating voltage of 5 kV and a current of 10 *μ*A in a microscope. The viability of the samples was improved by adding a gold sputter coating [22]. UV-Vis absorption spectroscopy of G-ZnO NPs in the wavelength range of 300–600 nm is performed using a twin beam PERKIN-ELMER spectrophotometer in a quartz cuvette with a path length of 1 cm and a resolution of 1 nm. For background correction, DDW is utilized as a reference [38].

#### 3.7.2. Statistical Analysis

Data were analyzed statistically employing the Duncan multiple range test (DMRT) using a full-randomized block design in R. (version 2.14.1). Origin software (version 2019b (9.65)) was used for principal component analysis (PCA).

## 4. Results and Discussion

### 4.1. Structural Properties of Synthesized G-ZnO NPs

XRD is used to calculate the crystallinity of synthesized G-ZnO NPs samples and also a phase of the crystal of G-ZnO NPs samples, as illustrated in Figure 1. All diffracted peaks are entirely matched to the normal peaks, according to ICDD data (card number: 080–0075). The hexagonal wurtzite structure characteristic of the G-ZnO NPs sample is presented, with *a* and *b* = 3.24 and *c* = 5.20, where *c*/*a* = 1.60. The G-ZnO NPs sample is obtained in a one step, according to the XRD pattern. The shape of the peaks reflects the lower size and crystalline nature of the samples. There are no peaks other than the normal peaks, indicating that the G-ZnO NPs produced are impurity free [22]. The nature of the shape of the peaks shows how the synthesized G-ZnO NPs are more crystalline and smaller in size. The highest peak was observed across the (101) orientation, at 2*θ* equal to 36.2° [23]. A pure wurtzite structure of ZnO is also supported by the peaks found at planes (100), (002), (102), (110), and (103) (stated in the ICDD card no. 080–0075, The International Centre for Diffraction Data, PA, USA). Three crystal lattice configurations of ZnO are known to exist: wurtzite (B4), cubic zinc-blende (B3), and rock salt (B1) [39, 40]. Only heteroepitaxial formation on cubic platforms, such as ZnS, GaAs/ZnS, and Pt/Ti/SiO2/Si, can maintain the zinc-blende type, whereas elevated pressure is required to produce the metastable rock salt or Rochelle salt (NaCl) form. With [0 0 0 1] or the basal plane as perhaps mainly often employed surface for development, wurtzite ZnO is a hexagonal structure with parameters “*a*” and “*c*” and a lattice constant (*c*/*a*) of $\sqrt{8/3}$ (1 : 633 in an ideal wurtzite hexagonal configuration) [41]. This structure is noncentrosymmetric and belongs to the space group C^4^_6v_ in Schoenflies notation and P6_3_mc in Hermann–Mauguin systems (a state in which space groups lack an inversion center) [41]. At normal temperatures, merely wurtzite structure contains a hexagonal unit cell that is thermodynamically stable, where each Zn atom in a tetrahedral structure is surrounded by four oxygen atoms and vice versa [39, 42].

X-ray dispersive energy spectrometry (EDX) is used to assess the chemical structure and quality of produced G-ZnO NPs samples, as shown in Figure 2. According to the EDX spectrum, the produced G-ZnO NPs samples included zinc and oxygen (also shown quantitatively in the figure as weight %). The background also shows the electron image of the sample used for analysis [22]. The availability of a substrate on which the G-ZnO NPs sample was held during instrumentation may account for the occurrence of a few additional peaks in comparison to the Zn and O peaks.

### 4.2. Morphological Nature of G-ZnO NPs

SEM observations have shown that G-ZnO NPs crystals do exist (Figure 3). The G-ZnO NPs sizes and their lengths cum diameters appear to be like grass on performing the sol-gel process. When compared to the crystal diameters, this also indicated the extensive lengths; consequently, their mean aspect ratios would likewise reveal the length of grass-shape form NPs. In keeping with the earlier studies, the morphology achieved in the current investigation is the effect of 0.135 gm zinc acetate precursor in a predetermined solution [43]. Similarly, surface characterization is performed using TEM [22]. It is used to validate the features of surface morphology along with the synthesis of G-ZnO NPs in the nanoscale range. The TEM data perfectly matched the SEM observation in this case.

The abundance of a range of G-ZnO NPs single crystals composed of pointed grass shaped in one-dimension (1D) was discovered by TEM investigation (Figure 4). The G-ZnO NPs were observed to be in frames resembling grass shape, and the increased geometry of the pointed rods showed the emergence of a unique 1D G-ZnO NPs lattice. The generation of finer particles was achieved by lengthening the incubation time following synthesis while maintaining the very same temperature. In the scientific literature, several preparation techniques, such as the solution-precipitation technique, sol-gel technique, spray-pyrolysis, microwave-assisted technique, hydrothermal technique, and water-assisted synthesis, have been utilized. These methods have produced ZnONPs in a variety of shapes and sizes, including nanothorns, nanorods, nanoflowers, microspheres, and nanoprisms [18].

### 4.3. Optical Characteristics of G-ZnO NPs

UV-Visabsorption spectroscopy is utilized to learn the optical properties of G-ZnO NPs. For the background inaccuracies, DW is employed as the reference material. Around 357 nm (in the UV-A region), a broad, compact, and sharp band of absorption is formed that is devoid of any other peak points, which is a characteristic of the pure hexagonal wurtzite ZnO structure (Figure 5). Moreover, the intensity of the absorption peak is found to be larger during longer incubation times (>1-2 months). When the incubation time is increased, a minor shift in the max of the G-ZnO NPs absorption spectra is seen. This hypsochromic shift in G-ZnO NPs*λ* max during longer incubation periods is attributed to an increase in the G-ZnO NPs aspect ratio, which also impacts G-ZnO NPs absorbance. Our findings are consistent with the earlier research that the peak shifts depending on the shape and size of the crystal, the process temperature, process type, solvents used, and several other sample factors [18, 44]. Additionally, it was shown that extending the incubation time after synthesis while maintaining the temperature resulted in much higher absorption peak intensities.

### 4.4. l/d Ratios of G-ZnO NPs

The measured length (l) and diameter (d) readings of the desired l/d ratios of long grass-likeone-dimensional crystals are associated with the nature of variables used during the G-ZnO NPs synthesis, as evidenced by SEM pictures [45]. Increasing the incubation period after synthesis, while keeping the temperature constant, improves the aspect-ratio identity of the crystals (Figure 6) [22]. This is attributable to the reason that when the temperature and incubation duration varies, both the length and diameter of the G-ZnO NPs decline, but the proportion of diameter (d) reduction is significantly more than the length (l). All of this culminates in the production of G-ZnO NPs, which resemble long grass-like morphologies (by increasing the incubation period by constantly maintaining the ambient temperature line).

### 4.5. Growth Mechanism of G-ZnO NPs

Here, the growth of G-ZnO NPs along different directions, i.e., [000I]; [0IĪI]; and [0IĪ0] axes, resulted in long grass-likeone-dimensionalG-ZnO NPs crystals. According to the results, increasing the incubation duration after synthesis while maintaining the temperature constant causes the l/d aspect ratios of the G-ZnO NPs to increase in distinct directions, i.e., [000I]; [0IĪI]; and [0IĪ0] axes, as shown in Figure 6. However, the maximum growth is towards [000I] facets as compared to the different axis. This is perhaps due to the cationic surfactant; palmityl trimethyl ammonium bromide, acts as a stabilizer for binding more into the [0IĪI] and [0IĪ0] axes, hence brings amendments in free energy and finally inactivates the advancements towards this axis [22, 23]. The growth continues on a similar pattern of further increasing the incubation period after synthesis while keeping the temperature constant. This overall leads to a great difference in G-ZnO NPs' d/l ratios having great surface areas, which could play a vital role in the nematicidal activity against *M. incognita* on chickpeas. But still, some of the G-ZnO NPs do not follow this trend and growth along different axis occurs.

### 4.6. Nematicidal Effect of G-ZnO NPs on J2s of *M. incognita* (*In Vvitro*)

#### 4.6.1. Effect of Various Concentrations of G-ZnO NPs on J2s Hatching Inhibition of *M. incognita*

A direct-contact study was utilized to investigate the inhibition of *M. incognita* J2s hatching by various concentrations (250, 500, 750, and 1000 ppm) of G-ZnO NPs, and there was a notable difference between concentrations. A direct-contact experiment was used to determine inhibition in J2s hatching of *M. incognita* by different concentrations (250, 500, 750, and 1000 ppm) of G-ZnO NPs, and a significant difference was observed with concentrations, indicating that hatching inhibition was directly influenced by concentrations. All concentrations were found to be effective in reducing J2s hatching compared to the control (water). The inhibition of J2s hatching increased significantly as concentrations increased from 250 ppm to 1000 ppm. Among all the concentrations tested, 1000 ppm showed the highest inhibition in J2s hatching, whereas 250 ppm predicts the least inhibition after 3 days of the exposure period. Other concentrations (500 and 750 ppm) inhibited J2s hatching considerably.  Table 1 shows the individual inhibitory impact of different concentrations (250, 500, 750, and 1000 ppm) of G-ZnO NPs on J2s hatching after 3 days of the exposure period.

#### 4.6.2. Effect of Various Concentrations of G-ZnO NPs on J2s Mortality of *M. incognita*

The mortality of J2s was determined using a direct-contact approach at various concentrations (250, 500, 750, and 1000 ppm) of G-ZnO NPs, and the results predict a considerable influence depending on concentrations and exposure periods. All concentrations were found to be toxic to J2s of *M. incognita* at a certain level. Usually, J2 mortality increases as exposure periods and concentrations increase. All concentrations exhibited higher mortality of J2s at 36 hours of the exposure period as compared with 12 and 24 hours. The 1000 ppm was found to be highly toxic to J2 at 36 hours as compared to other 250, 500, and 750 ppm. However, 250 ppm also exhibited significant J2s mortality compared to the control (water). There is no J2s mortality observed in the control. The result indicates that all concentrations were highly toxic to J2s and caused mortality from 42.00% to 70.00% at 36 hours.  Table 2 displays the negative effect of G-ZnO NP at various concentrations (250, 500, 750, and 1000 ppm) on J2s of *M. incognita*. G-ZnO NPs were shown to be highly toxic to J2s at 36 hours (LC50-621.53 ppm), 24 hours (LC50-969.64 ppm), and 12 hours (LC50-1352.96 ppm), respectively (Table 3).

In this study, G-ZnO NPs act as natural nematicides and had been reported to effectively suppress RKN, *M. incognita*. *In vitro* studies exhibited that all applied concentrations (250, 500, 750, and 1000 ppm) of G-ZnO NPs caused J2s mortality and induce inhibition in the J2s hatch. In-vitro experiment predicts the strong nematicidal potential of G-ZnO NPs. G-ZnO NPs were also found to be safe, causing no phytotoxicity. Furthermore, nematicidal efficacy was directly proportional to G-ZnO NPs concentration. The incubation duration was also a key component. As we increase G-ZnO NPs concentration from 250 to 1000 ppm, J2s mortality and J2s hatching inhibition were also increased in successive ways. The nematotoxic effect of G-ZnO NPs on *M. incognita* may be caused by a variety of activities, including disturbance of many cellular systems including membrane permeability, production of ATP, and oxidative stress reaction [46, 47]. Nanoparticle-induced disruptions in the cellular architecture of nematodes may be responsible for the presumed validation of J2's mortality. Ma et al. [48] found that heavy metals harmed *Caenorhabditis elegans* by destroying the integrity of cell membranes and altering the cations linked with proteins. According to Akhter et al. [49], varied concentrations of copper NPs (50, 100, 200, 400, and 800 g/mL) caused J2s mortality and egg-hatching inhibition of *M. incognita* to a varying degree. Mohammed and Reda [50] reported that Verox and the zinc oxide nanomaterial efficiently suppressed the egg-hatching of root-knot nematode, *Meloidogyne* spp. Duraisamy et al. [51] found that synthesized Sg-ZnO nanorods were toxic to *M. incognita* J2s and had a significant growth-promoting result on tomato seed germination and seedling length. The outcome of the in vitro study suggests that G-ZnO NPs affect directly or indirectly egg masses and J2s of *M. incognita*.

#### 4.6.3. Nematicidal Effect of G-ZnO NPs against *M. incognita*In-Planta Trial

In the pot experiment, different concentrations, viz., 250, 500, 750, and 1000 ppm, of G-ZnO NPs significantly decreased the galls and J2s in the soil and consequently enhanced the growth and photosynthetic pigments of chickpea as compared to only nematode-inoculated plants (J2s only).

#### 4.6.4. Effect on Growth Parameters

The results revealed that G-ZnONPs-treated plants thrived and developed faster than nematode-infected plants. Plant length and fresh weight showed significant differences (*p* ≤ 0.05) between G-ZnO NPs treated and only nematode-infested plants. The application of G-ZnO NPs @10 ml at various concentrations (250, 500, 750, and 1000 ppm) enhanced growth attributes, viz., the plant length and fresh weight significantly. The highest plant length and fresh weight were reported for those plants treated with 1000 ppm of G-ZnO NPs. It was followed by 750 ppm and 500 ppm. Furthermore, as compared to only J2s inoculated plants, plants treated with 250 ppm also showed significant improvement in the plant length and fresh weight. On the other hand, all the concentrations (250, 500, 750, and 1000 ppm) applied @10 ml were found to increase the number of pods and nodules as compared to only J2s-inoculated plants. Among all the concentrations applied, the 1000 ppm of G-ZnO NPs created additional prominence in increasing the number of pods and nodules/plants. It was followed by 750 ppm and 500 ppm. However, the lowest number of pods and nodules/plant was found in 250 ppm as compared to only J2s-inoculated plants. The improvement in growth parameters of chickpeas by the application of various concentrations of G-ZnO NPs is given in Figure 7.

#### 4.6.5. Effect on Photosynthetic Pigments

Application of G-ZnO NPs @10 ml of varying concentrations (250, 500, 750, and 1000 ppm) also showed significant improvement in the chlorophyll and carotenoid contents in the same way as in the case of growth parameters. The highest chlorophyll and carotenoid contents were reported for those plants treated with 1000 ppm of G-ZnO NPs. It was followed by 750 ppm and 500 ppm. However, the lowest chlorophyll and carotenoid contents were observed in those plants treated with 250 ppm as compared to only J2s inoculated plants. The individual enhancement in the chlorophyll and carotenoid contents of plants by various concentrations of G-ZnO NPs is given in Figure 8.

#### 4.6.6. Effect on J2s Population and Galls

The application of 10 ml of various concentrations of G-ZnO NPs inhibited *M. incognita* infection in respect of the population of J2s and galls/plant, and a significant difference was found between the concentrations when compared to only J2s-inoculated plants. At 1000 ppm, G-ZnO NPs achieved the highest reduction in galls and J2s population followed by 750 ppm, 500 ppm, and 250 ppm compared to only J2s-inoculated plants. The individual suppressive effect in the J2s population and galls by various concentrations of G-ZnO NPs is given in Figure 9. The outcome of the principal component analysis showed that the J2s population of *M. incognita* in soil and galls/plant was closely linked with various growth and photosynthetic metrics of chickpea. Scatter biplot analysis showed that applying 10 ml of varying concentrations (250, 500, 750, and 1000 ppm) of G-ZnO NPs effectively inhibited *M. incognita* infestation and improved chickpea development parameters (Figure 10).

The outcome of the present study established that G-ZnO NPs might be useful in the control of *M. incognita* on chickpeas. Furthermore, G-ZnO NPs applied at various concentrations significantly inhibit the infectivity incidence of J2s of *M. incognita* on chickpeas. The reduced nematode population and root galls were linked either with distraction in J2s entrance in chickpea roots or a halt in the progress of J2s that did pierce roots. G-ZnO NPs possess nematicidal potential which may deliver as a substitute for chemical nematicides that created environmental toxicity after repeated use. This study explored a substitute approach to be utilized in conjunction with the other current RKNs control methods. Our results also suggested that G-ZnO NPs directly or indirectly destroyed egg masses, caused J2s mortality, and induced resistance in chickpeas; so, we can assume that it can reduce the penetration of nematodes after treatment with different concentrations. The reduction in infectivity proportion increased if there was less attraction of J2s to roots and the absence of root exudates to attract nematodes by bionematicides [52]. Sharon et al. [53] revealed that the physical structure (e.g., size, shape, and homogeneity) of bioformed Ag-NPs was linked to their inhibitory effect, which likely played a significant part in nematode egg cell wall penetration and subsequent cell malfunction. Ag-NPs are not species-specific in their toxicity; and they may be used to control a variety of plant-parasitic nematodes and plant-pathogenic fungi. The mechanism of action of Ag-NPs is related to the disruption and dysfunction of various cellular systems in both eukaryotic and prokaryotic cells, including membrane permeability, ATP generation, and physiological response to oxidative stress [47, 54]. Algae-synthesized ZnO NPs demonstrated their positive effect on RKN management and nematode community suppression in soil and roots and may contribute in the suppression of *M. incognita* and have a significant impact on banana health [15]. When utilized to suppress the nematode infection of *M. incognita*, green-producedG-ZnO NPs had no plant phototoxicity. On the basis of the results, G-ZnO NPs have a great potential as a biostimulant component for plant development and as a method for controlling *M. incognita* on chickpea plants.

## 5. Conclusion

This study described the synthesis and characterization of novel long grass-likeone-dimensionalG-ZnO NPs crystals with the assistance of the sol-gel technique on further increasing the incubation period after synthesis while keeping the temperature constant. Their total effect on particle size, shape, and overall morphologies with l/d dimensions are stated. The SEM outcomes demonstrated the existence of G-ZnO NPs along different directions, i.e., [000I]; [0IĪI]; and [0IĪ0] axes occur Their average diameters range from 14 nm to 140 nm, and their lengths start from >500 nm, making their aspect-ratios start from 58. In conclusion, the growth pattern of the G-ZnO NPs indicated that the growth rate was greatest on [000I] facets. The presence of the palmityl trimethyl ammonium bromide complex (stabilizer) that binds more towards facets [0IĪI] and [0IĪ0] axis changes free energy and reduces the development of these aspects. Considerable UV-Vis light absorption by G-ZnO nanoparticles demonstrates their UV-A region activity (also called soft UV). The investigation led to the conclusion that G-ZnO NPs improved the growth characteristics and yields of chickpeas and decreased *M. incognita* infection. In addition, the study showed J2s mortality by G-ZnO NPs and their subsequent inhibition in J2s emergence of *M. incognita* (*in vitro*). This indicates an encouragement and recommendations for future research towards the beneficial role of G-ZnO NPs in enhancing various plant growth parameters grown in nematode-infected soil and their application in the biological control of *M. incognita* as a novel class of multifunctional nano-nematicide.

## Figures and Tables

**Figure 1:** X-ray diffraction (XRD) pattern of synthesized G-ZnO NPs via the sol-gel process.

**Figure 2:** EDX and quantitative analysis of the G-ZnO NPs along with its electron image (background).

**Figure 3:** SEM photograph of synthesized G-ZnO NPs via the sol-gel process.

**Figure 4:** TEM photograph of synthesized G-ZnO NPs via the sol-gel process.

**Figure 5:** UV-vis spectra of G-ZnO NPs.

**Figure 6:** Comparative chart showing length (l), diameter (d), and aspect-ratio (l/d) of long grass like one-dimensionalG-ZnO NPs crystals produced by extending the incubation period while keeping the ambient temperature line constant.

**Figure 7:** Effect of various concentrations (250, 500, 750, and 1000 ppm) of G-ZnO NPs on the growth attributes of chickpea.

**Figure 8:** Effect of various concentrations (250, 500, 750, and 1000 ppm) of G-ZnO NPs on the physiological attributes of chickpea.

**Figure 9:** Effect of various concentrations (250, 500, 750, and 1000 ppm) of G-ZnO NPs on the pathological attributes of chickpea.

**Figure 10:** The biplots of principal component analysis comparing the effect of various concentrations (250, 500, 750, and 1000 ppm) of G-ZnO NPs on various studied parameters of chickpea infected with *M. incognita*. PL: plant length; PFW: plant fresh weight; NOP: number of pods; NON: number of nodules; CHL: chlorophyll content; CRT: carotenoid content; GL = gall per plant; NP: nematode population in the 200 g soil sample.

**Table 1:** Effect of various concentrations of G-ZnO NPs on J2s hatching of *M. incognita in vitro* after 3 days.

Treatment	Exposure period (days)	Number of second-stage juveniles (mean ± SE) hatched in different concentrations (ppm)				
		1000	750	500	250	DW
G-ZnO NPs	3	115*e* ± 5.68 (72.61%)	139*d* ± 5.77 (66.90%)	170*c* ± 6.08 (5952%)	211*b* ± 6.08 (47.76%)	420*a* ± 0 (0%)

Each value is an average of five replicate, DW = distilled water (Control). Ppm: parts per million; SE: standard error. Values are given in parentheses represent percent inhibition in J2s hatching over the control. Values given without parentheses represent the number of the hatched J2s of *M. incognita* in different concentrations.

**Table 2:** Effect of various concentrations of G-ZnO NPs on the mortality of J2s of *M. incognita* after 12, 24, and 36 hours of the exposure period *in vitro*.

Treatment	Exposure period (hours)	Number of J2s dead in different concentrations (ppm)				
		1000	750	500	250	DW
G-ZnO NPs	12	47c ± 3.21 (42.72%)	32*d* ± 2.30 (29.09%)	20*c* ± 1.52 (18.18%)	10*d* ± 1.52 (9.09%)	0 ± 0 (0%)
	24	61*b* ± 3.78 (55.45%)	43*a* ± 3.05 (39.09%)	33*c* ± 2.08 (30%)	22*d* ± 2.64 (20%)	0 ± 0 (0%)
	36	77*ab* ± 3.46 (70%)	58*a* ± 3.21 (52.72%)	40*b* ± 3.46 (36.36%)	31*b* ± 2.08 (28.18%)	0 ± 0 (0%)

Each value is an average of five replicates, DW = distilled water (control). ppm: parts per million; SE: standard error. Values given in parentheses represent the percent J2s mortality over the control. Values given without parentheses represent the number of the dead J2s of *M*. *incognita* in different concentrations.

**Table 3:** Nematicidal activity of G-ZnO NPs against J2s of *M. incognita*.

Treatment	Exposure period (hours)	LC50 value in ppm (95% CL)
G-ZnO NPs	12	1352.96
	24	969.64
	36	621.53

LC_50_: lethal concentration caused 50% mortality after 12, 24, and 36 hours at 95% confidence limits. CL: confidence limit.

## Data Availability

The data used to support the findings of this study are included within the article.
